# A Case-Control Study on Risk Factors of Pulmonary Infection in Patients with Type 2 Diabetes Mellitus and Its Implications for Clinical Intervention

This article has been retracted.

**DOI:** 10.1155/2022/4492574

**Published:** 2022-04-12

**Authors:** Xue Li, Yanzi Ren, Ting Yan

**Affiliations:** Department of Endocrinology, The First People's Hospital of Jiangxia District, Wuhan City, 430200 Hubei Province, China

## Abstract

**Objective:**

To analyze the risk factors of pulmonary infection in patients with type 2 diabetes mellitus (T2DM) and its implications for clinical intervention.

**Methods:**

One hundred and twenty-five patients with type 2 diabetes treated in our hospital from January 2019 to November 2021 were divided into simple T2DM group (*n* = 80) and infection group (*n* = 45) according to whether they were complicated with pulmonary infection or not. Sputum samples of patients with infection were collected and identified by bacterial culture. The general conditions (age, sex, body mass index, course of disease, and length of stay), pulmonary complications (chronic bronchitis, emphysema, and obstructive pulmonary disease,), blood glucose control (fasting blood glucose and glycosylated hemoglobin), and treatment (use of hormones and antibiotics and invasive operation) were compared between the two groups. Univariate and multivariate analyses were used to screen the risk factors of pulmonary infection in patients with T2DM.

**Results:**

A total of 45 patients were found to be infected in this study. 68 pathogenic bacteria were detected in the sputum samples, of which 42 were Gram-negative (61.76%), 22 were Gram-positive (35.35%), and 4 were fungi (5.88%). Gram-negative bacteria were mainly Klebsiella pneumoniae, accounting for 25.00%, followed by Pseudomonas aeruginosa, Acinetobacter baumannii, and Escherichia coli. Gram-positive bacteria were mainly Staphylococcus aureus, accounting for 17.65%, followed by Streptococcus pneumoniae and Staphylococcus haemolyticus. The main fungi were Candida albicans (4.41%). The age, the course of T2DM, and the duration of hospitalization in the coinfection group were significantly higher than those in the T2DM group (*P* < 0.05). There was no significant difference in other indexes (*P* > 0.05). The number of patients with chronic bronchitis, emphysema, and obstructive pulmonary disease in the coinfection group was significantly higher than that in the T2DM group. The fasting blood glucose and glycosylated hemoglobin in the coinfection group were significantly higher than those in the T2DM group. The number of patients using hormone and antimicrobial agents and invasive operation in the coinfection group was higher than that in the simple T2DM group, and the difference was statistically significant (*P* < 0.05). Multivariate analysis showed that age, course of T2DM, length of hospital stay, complicated pulmonary disease, glycosylated hemoglobin, use of hormones and antibiotics, and invasive operation were all risk factors of pulmonary infection in patients with T2DM (*P* < 0.05).

**Conclusion:**

Gram-negative bacteria are the main pathogens of T2DM complicated with pulmonary infection. Drug sensitivity test should be combined to understand the drug resistance of pathogenic bacteria and use drugs reasonably to patients. Among them, advanced age, long course of T2DM, long hospital stay, complicated pulmonary disease, high level of glycosylated hemoglobin, use of hormones and antibiotics, and invasive operation were all risk factors of pulmonary infection in patients with T2DM. In clinical treatment, under the premise of using insulin to control blood sugar in an appropriate range, antibiotics should be used reasonably, pulmonary complications should be treated actively, pulmonary ventilation function should be improved, and invasive operation should be avoided as far as possible, which can effectively prevent the occurrence of T2DM complicated with pulmonary infection.

## 1. Introduction

With the rapid economic development and the acceleration of industrialization, the threat of noncommunicable diseases to human health is increasing day by day, in which diabetes and subsequent complications are ruthless killers to health. According to the International Diabetes Federation (IDF), there were 151 million people living with diabetes worldwide in 2000, and this year, the number has increased to 285 million. At the current rate of growth, it is estimated that nearly 500 million people will suffer from diabetes by 2030. The number of people with diabetes in China accounts for one of the largest number of people in the world. The 2008 survey showed that among adults over 20 years old, the prevalence rate of age-standardized diabetes was 9.7%, while the proportion of prediabetes was as high as 15.5%. This is equivalent to one in four adults with hyperglycemia. What is more serious is that 60.7% of the patients with diabetes in our country have not been diagnosed and cannot carry out effective treatment and education as soon as possible [1].

The chronic complications of diabetes pose a great threat to the life and quality of life of patients and bring heavy economic burden to the family and individual patients. 11.6% of the world's health care costs were spent on diabetes prevention and treatment in 2010, and the World Health Organization estimates that China's economic losses caused by diabetes and related cardiovascular diseases amounted to US $557.7 billion between 2005 and 2015. However, due to the complex pathogenesis of diabetes, human beings have not yet found a radical cure, which means that patients need to be treated for life [2].

Type 2 diabetes mellitus (T2DM) is a group of chronic metabolic diseases characterized by hyperglycemia, which can lead to multiple organ function damage (especially kidney, heart, peripheral nerves, blood vessels, eyes, etc.) [3]. Some studies have pointed out that in T2DM patients, the adhesion, chemotaxis, and phagocytosis of polymorphonuclear leukocytes may be impaired, and the function of cells involved in bactericidal activity in the antioxidant system may also be suppressed. Therefore, compared with non-T2DM patients, T2DM patients are more likely to suffer from various infectious diseases, among which the incidence of pulmonary infection is higher, which is one of the important factors leading to hospitalization and death of T2DM patients [4, 5]. Therefore, finding the risk factors of pulmonary infection in patients with T2DM and implementing preventive measures according to the risk factors are of great significance to reduce the pulmonary infection rate, improve the quality of life, and reduce the mortality. The purpose of this study was to explore the risk factors of pulmonary infection in patients with T2DM and analyze its implications for clinical intervention.

## 2. Patients and Methods

### 2.1. Participants' Information

A total of 125 patients with T2DM treated in our hospital from January 2019 to November 2021 were divided into diabetes group (*n* = 80) and infection group (*n* = 45). Inclusion criteria are as follows: (1) according to the diagnostic criteria of T2DM in China T2DM Prevention and treatment Guide [6] issued by the T2DM Branch of Chinese Medical Association in 2013: patients with typical diabetic symptoms (polydipsia, polyuria, and weight loss) and random blood glucose ≥11.1 mmol/L, fasting blood glucose (FPG) ≥7.0 mmol/L and blood glucose ≥11 mmol/L 2 hours after glucose load. (2) Diagnostic criteria of pulmonary infection: in accordance with the criteria of pulmonary infection established by the Respiratory Branch of the Chinese Medical Association [7] and in accordance with the new patchy infiltration, lobar or segmental consolidation, ground glass shadow, or interstitial changes, with or without pleural effusion, including any of the following four items: (1) the characteristics of lung consolidation and/or wet rale; (2) fever; (3) worsening symptoms of recent cough, expectoration, or original respiratory diseases, with or without purulent sputum, chest pain, dyspnea, and hemoptysis; (4) significant increase of white blood cells (>10 ×109/L) or significant decrease (<4×109/L), with or without nuclear left shift; and (3) the patient and his family members have informed consent and signed the informed consent form. Exclusion criteria are as follows: (1) patients with pulmonary tuberculosis, lung tumors, and other diseases; (2) patients with type 1 diabetes; (3) patients with dysfunction or malignant tumors of other important organs (kidney and liver); (4) patients with acute infection and severe inflammation within one month; and (5) patients during pregnancy and lactation.

### 2.2. Treatment Method

All patients were treated according to T2DM routine methods, such as insulin or oral hypoglycemic drugs according to their condition, daily dynamic monitoring of blood glucose concentration combined with reasonable diet and exercise improvement, and control of other complications.

### 2.3. Observation Index

Sputum samples of patients with infection were collected and identified by bacterial culture. The general conditions (age, sex, body mass index, course of disease, length of stay, smoking history, and drinking history), pulmonary complications and complications (chronic bronchitis, emphysema, obstructive pulmonary disease, and hypertension), blood glucose control (fasting blood glucose and glycosylated hemoglobin), and treatment (hormone and antimicrobial use and invasive operation) were collected from the two groups (age, sex, body mass index, course of disease, length of stay, and history of smoking and drinking), pulmonary complications and complications (chronic bronchitis, emphysema, obstructive pulmonary disease, and hypertension).

#### 2.3.1. Sputum Sample Detection

After rinsing the mouth, the patient needs to cough up the sputum into a sterile, dry sputum cup. Sputum samples need to be sent to the hospital microbiology unit for smear and microscopic examination within 2 hours. If the squamous epithelial cell count is less than 10 and the leucocyte count is greater than 25, or if the squamous epithelial cell count is less than 1 and the leucocyte count is less than 1.5, the sputum sample is judged to be satisfactory. The qualified sputum samples were isolated and cultured in the pathogen laboratory according to the relevant requirements of the National Operating Rules for Clinical Examination. The cultured pathogens were analyzed by automatic microbiological identification instrument (model: DW-M80, Hangzhou Great Microbiology). Quality control strains (Clinical Test Center of Ministry of Health) are the following: Pseudomonas aeruginosa (ATCC15442), Acinetobacter baumannii (ATCC19606), Escherichia coli (ATCC25922), Klebsiella pneumoniae (ATCC700603), Streptococcus pneumoniae (ATCC49619), Staphylococcus aureus (ATCC27217), Staphylococcus haemolyticus (ATCC31874), Candida albicans (ATCC10231), and Aspergillus (ATCC16865).

#### 2.3.2. Blood Glucose Detection

The fasting peripheral venous blood 4 mL was collected in the early morning, and the heparin anticoagulant tube was placed at room temperature for 30 minutes. The serum was separated after centrifugation at the speed of 4000 r/min for 15 minutes. Fasting blood glucose was measured by automatic biochemical analyzer, and glycosylated hemoglobin level was measured by automatic glycosylated hemoglobin analyzer.

### 2.4. Statistical Analysis

Using SPSS20.0 statistical software, before statistical analysis, the measurement data were tested by normal distribution and variance homogeneity analysis to meet the requirements of normal distribution or approximate normal distribution, expressed as $\bar{x}\pm \text{s}$. *t* test was used to compare the two groups, single factor analysis of variance was used to compare the mean of multiple groups, and *χ*^2^ test was used to represent the counting data with an example of *n* (%). Univariate and multivariate analyses were used to screen the risk factors of pulmonary infection in patients with T2DM (*P* < 0.05).

## 3. Results

### 3.1. The Status of Pathogens in Patients with Coinfection

A total of 45 patients were found to be infected in this study. 68 pathogenic bacteria were detected in the sputum samples, of which 42 were Gram-negative (61.76%), 22 were Gram-positive (35.35%), and 4 were fungi (5.88%). Gram-negative bacteria were mainly Klebsiella pneumoniae, accounting for 25.00%, followed by Pseudomonas aeruginosa, Acinetobacter baumannii, and Escherichia coli. Gram-positive bacteria were mainly Staphylococcus aureus, accounting for 17.65%, followed by Streptococcus pneumoniae and Staphylococcus haemolyticus. The main fungi were Candida albicans (4.41%). The distribution and composition of pathogens is shown in Table 1.

### 3.2. Comparison of General Conditions between the Two Groups of Patients

The age, the course of T2DM, and the duration of hospitalization in the coinfection group were significantly higher than those in the T2DM group (*P* < 0.05). There was no significant difference in other indexes (*P* > 0.05). All the data is presented in Table 2.

### 3.3. Comparison of Pulmonary Complications between the Two Groups

The number of patients with chronic bronchitis, emphysema, and obstructive pulmonary disease in the coinfection group was significantly higher than that in the T2DM group. All the data is presented in Table 3.

### 3.4. Comparison of Blood Glucose between the Two Groups

The fasting blood glucose and glycosylated hemoglobin in the coinfection group were significantly higher than those in the T2DM group. All the data is presented in Table 4.

### 3.5. Comparison of Treatment between the Two Groups

The number of patients using hormone and antimicrobial agents and invasive operation in the coinfection group was higher than that in the simple T2DM group, and the difference was statistically significant (*P* < 0.05). All the data is presented in Table 5.

### 3.6. Multivariate Analysis of Pulmonary Infection in Patients with T2DM

Multivariate analysis showed that age, course of T2DM, length of hospital stay, complicated pulmonary disease, glycosylated hemoglobin, use of hormones and antibiotics, and invasive operation were all risk factors of pulmonary infection in patients with type 2 diabetes mellitus (*P* < 0.05). All the data is presented in Table 6.

## 4. Discussion

T2DM is a chronic disease with increased blood glucose levels due to insufficient insulin secretion and/or insulin resistance caused by genetic and/or environmental factors. The disease can cause multisystem damage, resulting in eye, kidney, nerve, heart, blood vessels, and other tissue and organ dysfunction [8]. The prevalence rate of diabetes is increasing rapidly all over the world, especially in developing countries. Diabetes has become the most important endocrine and metabolic disease in clinic, and it is also one of the most important chronic noncommunicable diseases advocated by the United Nations in the world [9]. The prevalence rate of T2DM in China is 10.4%. The prevalence rates of men and women are 11.1% and 9.6%, respectively, and the prevalence rate of men is higher than that of women [10]. The etiology of T2DM is not clear. Generally speaking, it is caused by both genetic and environmental factors. The main pathogenesis is pancreatic beta-cell dysfunction and insulin resistance, while pancreatic alpha-cell dysfunction and lack of intestinal secretory hormones also play an important role [11].

Patients with hypertension and dyslipidemia have an increased risk of T2DM. Among these environmental factors, obesity occupies a central position, because it is not only the result of many environmental factors but also may be the cause of multiple environmental factors [12]. At present, it is believed that the main pathogenesis of T2DM includes insulin resistance: the main mechanisms of insulin-reducing hypoglycemia include inhibiting glucose production in liver, stimulating glucose uptake in visceral tissue (such as liver), and promoting glucose utilization in peripheral tissue (skeletal muscle and fat). Insulin resistance refers to the reduced sensitivity of the target organs to insulin, that is, insulin levels may be sufficient but cannot effectively act on the target organs. Defective *β*-cell function makes insulin production insufficient to compensate for the effects of insulin resistance, which is the final link in the pathogenesis of T2DM. [12]. In patients with T2DM, the number of islet *β*-cells decreased significantly, and the sensitivity of *α* cells to glucose decreased, which led to the increase of glucagon secretion and liver glucose output [13]. Deficiency of enteropogon secretion: GLP-1 is secreted by the intestine, and the main biological functions are the stimulating *β*-cell growth, secretion of insulin, and inhibiting glucagon secretion. Other biological effects include delaying the emptying of gastric contents, inhibiting appetite and food intake, and promoting the increase of *β*-cells [14]. The GLP-1 of T2DM patients is lower than that of normal subjects after eating, which leads to insufficient insulin secretion and increase of blood glucose [14, 15].

Pulmonary infection ranks first in infectious complications, which is one of the important causes of death in patients with diabetes [16]. The study found that the reason why diabetic patients are prone to pulmonary infection is that the plasma osmotic pressure of the body increases under the condition of hyperglycemia, which slows down the division speed of lymphocytes, weakens the phagocytosis of leukocytes, and decreases the immune function, which provides favorable conditions for the growth of bacteria [16]. Hyperglycemia can also lead to acidosis, hyperosmotic diuresis, and other complications, which are often associated with electrolyte disorders and acid-base imbalance [17]. Disturbances in sugar, protein, and fat metabolism in diabetics are one of the main causes of lung infections [18]. In addition, the synthesis of bacterial enzymes in alveolar macrophages decreased, and fatty acid deficiency and disease resistance greatly decreased [19]. Moreover, diabetes is a chronic lifelong disease with a long course of disease, which creates conditions for the invasion and reproduction of bacteria, and is more prone to lung infection [20]. By collecting a number of data of patients with T2DM, our current study screened the risk factors of pulmonary infection and analyzed the significance of clinical intervention.

A total of 45 patients were found to be infected in this study. 68 pathogenic bacteria were detected in the sputum samples, of which 42 were Gram-negative (61.76%), 22 were Gram-positive (35.35%), and 4 were fungi (5.88%). Gram-negative bacteria were mainly Klebsiella pneumoniae, accounting for 25.00%, followed by Pseudomonas aeruginosa, Acinetobacter baumannii, and Escherichia coli. Gram-positive bacteria were mainly Staphylococcus aureus, accounting for 17.65%, followed by Streptococcus pneumoniae and Staphylococcus haemolyticus. The main fungi were Candida albicans (4.41%). It is suggested that the main pathogens in patients with type 2 diabetes mellitus complicated with pulmonary infection are Gram-negative bacteria. In clinical studies, some scholars have found that pulmonary microvascular lesions may occur in patients with T2DM, which will lead to oxygen diffusion disturbance, induce lung tissue hypoxia, and further weaken the immune function of the patient [21]. High sugar also promotes the multiplication of pathogens, which can easily multiply in the patient's lungs and lead to pneumonia. At present, the clinical treatment of simple pneumonia is mainly based on antimicrobial therapy. However, the immunity of patients with T2DM is relatively low, which can easily lead to the increase of drug resistance of pathogens, and the treatment of T2DM with pulmonary infection is more complicated than that of common pneumonia. Therefore, the treatment of patients with T2DM complicated with pulmonary infection should first pass the detection of pathogenic microorganisms, analyze the distribution of pathogenic bacteria, combined with drug sensitivity test, understand the drug resistance of pathogenic bacteria, and then use drugs reasonably to the patients in order to reduce the mortality of T2DM complicated with acute pneumonia. In this study, the sputum samples of patients were collected to detect the pathogenic microorganisms, and the distribution of pathogenic bacteria was analyzed. According to the test results, the main pathogens of T2DM complicated with pulmonary infection were Gram-negative bacteria, which may be due to the relative increase of plasma osmotic pressure and the weakening of phagocytosis of monocytes, neutrophils, and macrophages in patients with T2DM under high glucose state [21]. According to the results of pathogen detection, Klebsiella pneumoniae, Pseudomonas aeruginosa, and Staphylococcus aureus are the main pathogens of T2DM complicated with acute pneumonia. It is suggested that clinicians should give priority to anti-Gram-negative bacteria in this kind of patients. Clinical workers should reduce the use of broad-spectrum antibiotics as much as possible, avoid the increase of drug resistance of pathogens caused by the abuse of antibiotics, and the production of superbacteria, so as to increase the difficulty and risk of follow-up clinical treatment [21].

Through univariate and multivariate analysis, it was found that age, course of T2DM, length of hospital stay, complicated lung disease, glycosylated hemoglobin, use of hormones and antibiotics, and invasive operation were all risk factors of pulmonary infection in patients with T2DM. There are a large number of normal bacteria in the pharynx of normal people, which maintain a certain balance. However, with the increase of age and the prolongation of the course of the disease, the functions of the respiratory system gradually decline, and the number of pathogenic bacteria living in the respiratory tract will increase, coupled with the decrease of mucociliary function in the trachea and bronchi of the elderly, resulting in poor cough reflex, the elasticity of lung tissue decreases progressively, sputum function decreases, bacteria are prone to invade the lower respiratory tract through the upper respiratory tract, and finally lead to lung infection [16]. The blood glucose level of elderly patients with diabetes has been at a high level for a long time, which creates a good living environment for the growth and development of pathogenic bacteria and is more likely to lead to pathogenic bacteria infection. Meanwhile, in the state of hyperglycemia, the plasma osmotic pressure of the body will increase accordingly, so that the division of lymphocytes can be delayed, thus inhibiting the function of neutrophils and mononuclear macrophages and reducing the resistance to pathogenic bacteria. In addition, most of the elderly patients with diabetes have hypoxemia, which reduces the blood volume in pulmonary capillaries and the content of pulmonary surfactant, which leads to the imbalance of blood flow and increases the probability of pulmonary infection. With the prolongation of hospitalization, the colonization proportion of multisite pathogens increased significantly, and the risk of cross-infection increased with the duration of hospitalization.

The following preventive measures are proposed to address the above risk factors: (1) minimize the length of hospital stay, as prolonged hospitalization increases the chances of lung infection in patients; (2) to keep the respiratory tract unobstructed, active measures should be taken for patients with pulmonary infection, such as tapping the patient's lungs, promoting sputum discharge, reducing the use of hormones, encouraging patients to move their limbs and giving sufficient water to the respiratory tract. Meanwhile, sputum samples should be taken from patients, targeted treatment for sputum infection bacteria can be carried out, and combined drugs can be taken if necessary; (3) to actively control blood sugar, as glycosylated hemoglobin is closely related to the occurrence of pulmonary infection, it is particularly important to monitor blood sugar. Furthermore, reasonable diet and exercise should be arranged to control blood sugar within an ideal range to reduce pulmonary infection [23]; (4) rational use of antibiotics and hormones, strict use of antibiotics, and targeted use of antibiotics with narrow antibacterial spectrum according to etiological culture, and (5) unnecessary invasive operation should be avoided as far as possible in the process of diagnosis and treatment of T2DM patients. Aseptic operation should be strictly carried out to shorten the indwelling time of all kinds of invasive catheters, so as to reduce the risk of pathogen infection.

Taken together, the main pathogens of T2DM complicated with pulmonary infection are Gram-negative bacteria, which should be combined with drug sensitivity test for use drugs reasonably to patients. Among them, advanced age, long course of T2DM, long hospital stay, complicated pulmonary disease, high level of glycosylated hemoglobin, use of hormones and antibiotics, and invasive operation were all risk factors of pulmonary infection in patients with T2DM. In clinical treatment, under the premise of using insulin to control blood sugar in an appropriate range, antibiotics should be used reasonably, pulmonary complications should be treated actively, pulmonary ventilation function should be improved, and invasive operation should be avoided as far as possible, which can effectively prevent the occurrence of T2DM complicated with pulmonary infection. Nevertheless, our study still had some shortcomings, such as the number of cases selected was not large enough and all were retrospective, so the conclusion of our study needs to be confirmed by future multicenter prospective studies with a larger number of cases.

## Figures and Tables

**Table 1:** Distribution and constituent ratio of pathogens in patients with T2DM complicated with pulmonary infection (%).

Pathogenic bacteria	Number of plants (*n* = 68)	Constituent ratio (%)
Gram-negative bacteria	42	61.76
Klebsiella pneumoniae	17	25.00
Pseudomonas aeruginosa	13	19.12
Acinetobacter baumannii	8	11.76
Escherichia coli	4	5.88
Gram-positive bacteria	22	35.35
Staphylococcus aureus	12	17.65
Streptococcus pneumoniae	7	10.29
Staphylococcus haemolyticus	3	4.41
Fungus	4	5.88
Candida albicans	3	4.41
Aspergillus	1	1.47

**Table 2:** Comparison of the general conditions of the two groups of patients [*n* (%), $\bar{x}\pm \text{s}$].

Data	*N*	Simple T2DM group (*n* = 80)	Combined infection group (*n* = 45)	*χ* ^2^/*t*	*P*
Gender					
Male	71	45 (63.38)	26 (36.62)		
Female	54	35 (64.81)	19 (35.19)	0.027	0.868
Age (year)	125	54.32 ± 12.26	65.79 ± 10.39	5.294	<0.001
T2DMCourse of disease	125	8.74 ± 2.36	5.62 ± 1.43	8.066	<0.001
Body mass index (kg/m^2^)	125	24.26 ± 2.28	24.17 ± 2.42	0.207	0.836
Smoking					
Yes	64	42 (48.76)	22 (32.23)		
No	61	38 (47.44)	23 (33.33)	0.150	0.698
Drink alcohol					
Yes	54	34 (62.96)	20 (37.04)		
No	71	46 (64.79)	25 (35.21)	0.044	0.833
Hospitalization time (*d*)	125	8.57 ± 2.64	17.78 ± 1.15	22.216	<0.001

**Table 3:** Comparison of pulmonary complications between the two groups [*n* (%)].

Group	*N*	Chronic bronchitis	Emphysema	Obstructive pulmonary disease
Simple T2DM group	80	6 (7.50)	3 (3.75)	10 (12.50)
Combined infection group	45	14 (31.11)	9 (20.00)	18 (40.00)
*t*		11.946	8.763	12.529
*P*		<0.001	0.003	<0.001

**Table 4:** Comparison of blood glucose between the two groups ($\bar{x}\pm \text{s}$).

Group	*N*	Fasting blood glucose (mmol/L)	Glycosylated hemoglobin (%)
Simple T2DM group	80	8.89 ± 1.69	9.12 ± 1.36
Combined infection group	45	11.55 ± 2.48	12.53 ± 2.71
*t*		7.106	9.369
*P*		<0.001	<0.001

**Table 5:** Comparison of treatment between the two groups [*n* (%)].

Group	*N*	Use of hormone	Use of antimicrobials	Perform intrusive operations
Simple T2DM group	80	20 (7.50)	13 (3.75)	7 (12.50)
Combined infection group	45	26 (31.11)	22 (20.00)	18 (40.00)
*t*		13.304	15.218	17.578
*P*		<0.001	<0.001	<0.001

**Table 6:** Multivariate analysis of pulmonary infection in patients with type 2 diabetes mellitus.

Factors	*β*	SE	wald*χ*^2^	OR	*P*	95% CI
Age	0.426	0.115	13.722	1.531	<0.001	1.222~1.198
Course of T2DM	0.559	0.158	12.517	1.749	<0.001	1.283~2.384
Hospitalization time	0.479	0.126	14.452	1.614	<0.001	1.261~2.067
Complicated with lung disease	0.638	0.216	8.724	1.893	0.003	1.239~2.890
Fasting blood glucose	0.518	0.347	2.229	1.679	0.136	0.850~3.314
Glycosylated hemoglobin	0.721	0.247	8.521	2.056	0.003	1.267~3.337
Hormone use	0.578	0.182	10.086	1.782	0.001	1.248~2.547
Use of antimicrobials	0.623	0.302	4.256	1.865	0.039	1.032~3.370
Perform intrusive operations	0.485	0.124	15.298	1.624	<0.001	1.274~2.071

## Data Availability

No data were used to support this study.

## References

[1] Chinese Elderly Type 2 Diabetes Prevention and Treatment of Clinical Guidelines Writing Group (2022). Clinical guidelines for prevention and treatment of type 2 diabetes mellitus in the elderly in China (2022 edition). *Zhonghua Nei Ke Za Zhi*.

[2] Schmidt A. M. (2018). Highlighting diabetes mellitus. *Arteriosclerosis, Thrombosis, and Vascular Biology*.

[3] Henning R. J. (2018). Type-2 diabetes mellitus and cardiovascular disease. *Future Cardiology*.

[4] Haiyan Y., Yunxiu Y., Yunhua Y. (2021). Study on the relationship between serum SP-D expression, gene polymorphism and pulmonary infection in elderly patients with diabetic nephropathy. *Journal of Modern Laboratory Medicine*.

[5] Drucker D. J. (2020). Coronavirus infections and type 2 diabetes-shared pathways with therapeutic implications. *Endocrine Reviews*.

[6] Diabetic Branch of Chinese Medical Association (2013). Chinese guidelines for the prevention and treatment of type 2 diabetes mellitus (2013 edition). *Chinese Journal of Endocrine and Metabolism*.

[7] Respiratory Branch of Chinese Medical Association (2016). Guidelines for the diagnosis and treatment of pneumonia in Chinese adults (2016 Edition). *Chinese Journal of Tuberculosis and Respiration*.

[8] Hackett R. A., Steptoe A. (2017). Type 2 diabetes mellitus and psychological stress -- a modifiable risk factor. *Nature Reviews. Endocrinology*.

[9] Zimmet P., Alberti K. G., Magliano D. J., Bennett P. H. (2016). Diabetes mellitus statistics on prevalence and mortality: facts and fallacies. *Nature Reviews. Endocrinology*.

[10] Gao C., Sun X., Lu L., Liu F., Yuan J. (2019). Prevalence of gestational diabetes mellitus in mainland China: a systematic review and meta-analysis. *Journal of Diabetes Investigation*.

[11] Faselis C., Katsimardou A., Imprialos K., Deligkaris P., Kallistratos M., Dimitriadis K. (2020). Microvascular complications of type 2 diabetes mellitus. *Current Vascular Pharmacology*.

[12] Lehrke M., Marx N. (2017). Diabetes mellitus and heart failure. *The American Journal of Medicine*.

[13] Agashe S., Petak S. (2021). Cardiac autonomic neuropathy in diabetes mellitus. *Methodist DeBakey Cardiovascular Journal*.

[14] Meiqin W., Dongfang L., Bo B. (2020). Effects of novel enterotropic insulin analogues on inflammatory response to cerebral ischemia-reperfusion in diabetic rats. *Chinesse Journal of Geriatric Cardiovascular and Cerebrovascular Diseases*.

[15] Zongguo Z., Hongyu Y., Lan H. (2021). Correlation between serum microRNA-152 expression level and blood lipid metabolism and insulin resistance in patients with diabetes mellitus. *Chinese Journal of Modern Medicine*.

[16] Weipeng D., Haixia W., Man X. (2021). Characteristics of pathogens of pulmonary infection and its correlation with inflammatory factors and pulmonary function in patients with type 2 diabetes mellitus. *Chinese Journal of Pathogenic Biology*.

[17] Pipeleers L., Wissing K. M., Hilbrands R. (2019). Acid-base and electrolyte disturbances in patients with diabetes mellitus. *Acta Clinica Belgica*.

[18] Gougeon R., Morais J. A., Chevalier S., Pereira S., Lamarche M., Marliss E. B. (2008). Determinants of whole-body protein metabolism in subjects with and without type 2 diabetes. *Diabetes Care*.

[19] Kunxia X., Feng Z., Xiaoqiang F. (2021). Effects of vitamin A combined with insulin on the frequency and complications of glycosylated hemoglobin hypoglycemia in children with type 1 diabetes mellitus. *Maternal and Child Health Care in China*.

[20] Patel M. R. (2020). Social determinants of poor management of type 2 diabetes among the insured. *Current Diabetes Reports*.

[21] Ting L., Yayang Z., Jiangang W. (2020). Effects of different inhaled oxygen concentrations on perioperative pulmonary function in patients with diabetes mellitus complicated with microangiopathy. *Chinese Journal of Modern Surgery*.

[22] Saeedi P., Petersohn I., Salpea P. (2019). Global and regional diabetes prevalence estimates for 2019 and projections for 2030 and 2045: results from the International Diabetes Federation Diabetes Atlas. *Diabetes Research and Clinical Practice*.

[23] Nery C., Moraes S. R. A., Novaes K. A., Bezerra M. A., Silveira P. V. D. C., Lemos A. (2017). Effectiveness of resistance exercise compared to aerobic exercise without insulin therapy in patients with type 2 diabetes mellitus: a meta-analysis. *Brazilian Journal of Physical Therapy*.

